RETRACTED

# Dynamic Action of Carotenoids in Cardioprotection and Maintenance of Cardiac Health 

**DOI:** 10.3390/molecules17044755

**Published:** 2012-04-23

**Authors:** Mahesh Agarwal, Royapuram P. Parameswari, Hannah R. Vasanthi, Dipak K. Das

**Affiliations:** 1 Department of Biotechnology, School of Life Sciences, Pondicherry University, Puducherry-605014, India; Email: mhsh.agarwal@gmail.com (M.A.); hrvasanthi@gmail.com (H.R.V.); 2 Herbal & Indian Medicine Research Laboratory, Sri Ramachandra University, Chennai 600 116, India; Email: paramsarathy@gmail.com; 3 Cardiovascular Research Centre, School of Medicine, University of Connecticut, Farmington 06030-1110, CT, USA

**Keywords:** oxidative stress, ROS, RNS, antioxidants, carotenoids, cardiovascular disease

## Abstract

Oxidative stress has been considered universally and undeniably implicated in the pathogenesis of all major diseases, including those of the cardiovascular system. Oxidative stress activate transcriptional messengers, such as nuclear factor—κB, tangibly contributing to endothelial dysfunction, the initiation and progression of atherosclerosis, irreversible damage after ischemic reperfusion, and even arrhythmia, such as atrial fibrillation. Evidence is rapidly accumulating to support the role of reactive oxygen species (ROS) and reactive nitrogen species (RNS) as intracellular signaling molecules. Despite this connection between oxidative stress and cardiovascular disease (CVD), there are currently no recognized therapeutic interventions to address this important unmet need. Antioxidants that provide a broad, “upstream” approach via ROS/RNS quenching or free radical chain breaking seem an appropriate therapeutic option based on epidemiologic, dietary, and *in vivo* animal model data. Short-term dietary intervention trials suggest that diets rich in fruit and vegetable intake lead to improvements in coronary risk factors and reduce cardiovascular mortality. Carotenoids are such abundant, plant-derived, fat-soluble pigments that functions as antioxidants. They are stored in the liver or adipose tissue, and are lipid soluble by becoming incorporated into plasma lipoprotein particles during transport. For these reasons, carotenoids may represent one plausible mechanism by which fruits and vegetables reduce the risk of chronic diseases as cardiovascular disease (CVD). This review paper outlines the role of carotenoids in maintaining cardiac health and cardioprotection mediated by several mechanisms including redox signaling.

## 1. Introduction

Reactive oxygen species (ROS) and reactive nitrogen species (RNS) play important roles in regulation of cell survival. In general, moderate levels of ROS/RNS may function as signals to promote cell proliferation and survival, whereas severe increases of ROS/RNS can induce cell death. Under physiologic conditions, the balance between generation and elimination of ROS/RNS maintains the proper function of redox-sensitive signaling proteins. Normally, the redox homeostasis ensures that the cells respond properly to endogenous and exogenous stimuli. However, when the redox homeostasis is disturbed, oxidative stress may lead to aberrant cell death and contribute to disease development [1]. Oxidative damage by free radicals has been well investigated within the context of oxidant/antioxidant balance. Indeed, oxidative stress describes various deleterious processes resulting from an imbalance between the excessive formation of reactive oxygen and/or nitrogen species and limited antioxidant defenses [2]. In this regard, cardiovascular risk factors significantly cause oxidative stress, which contributes to a disruption in the balance between nitric oxide (NO) and reactive oxygen species, with a resulting relative decrease in NO bioavailability. The resulting endothelial dysfunction has been supposed to be the first step of atherosclerosis. Further, majority of cardiovascular diseases follow from complications of atherosclerosis. In addition, an important initiating event for atherosclerosis may well be the transport of oxidized low-density lipoprotein across the endothelium into the artery wall [3,4,5].

RETRACTED

In the post-ischemic myocardium, elevated levels of exogenous ROS are generated in cardiomyocytes, endothelial cells, and infiltrating neutrophils that can lead to cellular dysfunction and necrosis. ROS most likely contribute to the pathogenesis of myocardial infarction (MI) and serve as mediators of the reversible ventricular dysfunction (stunning) that often accompanies reperfusion of ischemic myocardium. Nutritional epidemiologic research demonstrates that those who consume higher amounts of fruits and vegetables tend to have lower rates of heart and vascular diseases, including coronary heart disease and stroke [6]. Carotenoids present in fruits and vegetables may prevent heart and vascular disease in a number of ways. The present review outlines the role of various carotenoids in cardiac health and cardioprotection mediated by several mechanisms including redox signaling.

## 2. Mechanisms of Redox Signaling

Redox signaling plays a pivotal role in many disorders—for example, vascular smooth muscle proliferation, atherosclerosis, angiogenesis, cardiac hypertrophy, fibrosis, remodeling [7]. ROS may induce acute (that is, over seconds to minutes) alterations in cellular functions via specific covalent modifications of target molecules. For example, key proteins involved in myocardial excitation-contraction coupling, such as sarcolemmal ion channels, sarcoplasmic reticulum calcium release channels, and contractile proteins, can all undergo redox sensitive alterations in activity [8]. ROS also exert important acute effects on cellular energetics. Chronic changes (that is, over hours and days) in cell phenotype result from modulation of intracellular signalling pathways, such as mitogen activated protein kinases (MAPKs), and redox sensitive transcription factors (for example, NF-kB, HIF-1, AP-1), with consequent alterations in gene and protein expression [9]. Specificity of signalling derives both from upstream ligand dependent stimulation of ROS production by different enzymatic sources and the targeting of specific downstream pathways by ROS. A wide variety of genes are redox sensitive through the above pathways, depending upon the context—for example, VCAM-1, MCP-1, PAI-1, and PDGF during endothelial cell activation [7].

RETRACTED

## 3. Antioxidants in Redox Status

In recent years there is an upsurge in the areas related to newer developments in prevention of disease especially the role of free radicals and antioxidants. ‘Antioxidants’ are substances that neutralize free radicals or their actions. Nature has endowed each cell with adequate protective mechanisms against any harmful effects of free radicals: superoxide dismutase (SOD), glutathione peroxidase, glutathione reductase, thioredoxin, thiols and disulfide bonding are buffering systems in every cell. α-Tocopherol (vitamin E) is an essential nutrient which functions as a chain-breaking antioxidant which prevents the propagation of free radical reactions in all cell membranes in the human body. Ascorbic acid (vitamin C) is also part of the normal protecting mechanism. Other non-enzymatic antioxidants include carotenoids, flavonoids and related polyphenols, α-lipoic acid, glutathione etc [10].

## 4. Carotenoids as Redox Agents

There is evidence to suggest that carotenoids act as modulators of intracellular redox status. Their ability to function as antioxidants has been known for many years. They are not just “another group of natural pigments”, they are substances with very special and remarkable properties that no other group of substances possess and that form the basis of their many, varied functions and actions in all kinds of living organisms. The conjugated double bond structure is primarily responsible for the ability of β-carotene to quench singlet oxygen physically without degradation, and for the chemical reactivity of β-carotene with free radicals such as the peroxyl, hydroxyl, and superoxide radicals. Carotenoids have been shown to be able to prevent or decrease oxidative damage to DNA, lipid and proteins [11,12].

RETRACTED

Conversely, according to Amengual *et al*., carotenoids can impair respiration and induce oxidative stress in β,β-carotene-9',10'-oxygenase (BCDO2)-deficient mice and in human cell cultures [13] possibly acting as pro-oxidants and increasing the total radical yield in a system [14]. The key factor to determine the switch of carotenoids from antioxidant to pro-oxidant is the oxygen partial pressure (pO_2_) and the carotenoid concentration [15,16]. At higher pO_2_ a carotenoid radical can react with molecular oxygen to generate a carotenoid- peroxyl radical which can act as pro-oxidant by promoting oxidation of unsaturated lipids. 

### 4.1. Structure of Carotenoids

The carotenoids are isoprenoid compounds, biosynthesized by tail-to-tail linkage of two C_20_ geranylgeranyl diphiosphate molecules. This produces the parent C_40_ carbon skeleton from which all the individual variations are derived. The carotenoids basic structure and numbering scheme is illustrated in Figure 1. The most striking and characteristic feature of carotenoid structure is the long stem of alternate single and double bonds that forms the central part of the molecule. This constitutes a conjugated system in which the п-electrons are effectively delocalized over the entire length of the polyene chain. It is the feature that gives the carotenoids as a group their distinctive molecular shape, chemical reactivity and light absorbing properties [17]. Among the natural and synthetic carotenoids carrying different 5- and 6-membered ring substituents at the end of the conjugated double bond system, the location and nature of the substituent at the 6-membered ring had little influence on the activity of different carotenoids [18]. Further, the activity of carotenoids differs depending upon the size of ring substituents.

**Figure 1:** Basic chemical structure of carotenoids.

### 4.2. Bioavailability and Metabolism of Carotenoids

Several factors influence the absorption of carotenoids. Food processing and cooking that cause mechanical breakdown of the tissue releasing the carotenoids improves their absorption [19,20,21]. They are absorbed into the gastrointestinal mucosal cells and appear unchanged in the circulation and tissues [20,21,22]. In the intestine the carotenoids are absorbed by passive diffusion after being incorporated into the micelles that are formed by dietary fat and bile acids. The micellular carotenoids are then incorporated into the chylomicrons and released into the lymphatic system. They are then incorporated into the lipoprotein at the site of the liver and released into the blood stream. Carotenoids are absorbed differentially by different tissues. The major site of tissue storage of carotenoids is the adipose tissue [22,23].

RETRACTED

## 5. Cardioprotective Mechanisms of Carotenoids

### 5.1. Antioxidant Activity

Oxidative stress and free radical attack on biological structures are believed to be major factors in the initiation and propagation of the development of many degenerative diseases. In general, carotenoids behave as effective antioxidants *in vitro* [24,25] and clear evidence exists from a majority of epidemiological studies on the incidence of CVD indicating an inverse relationship with dietary carotenoids [26] and circulating carotenoid levels. Carotenoids may function as chain breaking antioxidants reducing lipid peroxidation of such vulnerable membranes. The antioxidant properties of carotenoids are primarily associated with their ability to quench singlet oxygen [27,28] and scavenge free radicals [29,30,31,32]. In carotenoids the conjugated carbon double-bond system is considered to be the single most important factor in energy transfer reactions, such as those found in photosynthesis [33]. It is this feature of the molecule that also permits the quenching of singlet oxygen (^1^O_2_). *In vitro* studies have shown that carotenoids are efficient quenchers of singlet oxygen, directly scavenge free radicals, and inhibit lipid peroxidation [34]. They exhibit considerable differences in the rate of quenching singlet oxygen, with lycopene having the strongest quenching ability of those studied, followed by α-carotene, β-carotene, zeaxanthin, lutein, and β-cryptoxanthin [35]. Lycopene has significant antioxidant potential *in vitro* and has been hypothesized to play a prominent role in preventing CVD [36,37,38]. In this sense, the antioxidant activity of some carotenoids during radical peroxide-induced cholesterol oxidation was investigated by Palozza and co-workers [39], showing that carotenoids exerted a significant antioxidant activity, in the decreasing activity order indicated: astaxanthin, cantaxanthin, lutein and β-carotene. Astaxanthin and canthaxanthin are scavengers of free radicals, chain-breaking antioxidants and potent quenchers of reactive oxygen and nitrogen species including singlet oxygen, single and two electron oxidants [40,41,42]. They (astaxanthin and canthaxanthin) have terminal carbonyl groups that are conjugated to a polyene backbone [42] and are more potent antioxidants and scavengers of free radicals than carotene carotenoids such as β-carotene [42,43,44]. For these reasons dietary supplementation with astaxanthin has the potential to provide antioxidant protection of cells and from atherosclerotic cardiovascular disease [45]. McNulty *et al*., studied the differential effects of carotenoids on lipid peroxidation due to membrane interactions. The results indicated that the distinct effects of carotenoids on lipid peroxidation are due to membrane structure changes [46]. These contrasting effects of carotenoids on lipid peroxidation may explain differences in their biological activity. Wilhelmstahl *et al*., have stated that the ring system of the carotenoids plays a role with respect to biological effects on intracellular communication [47].

RETRACTED

### 5.2. Hypocholesterolemic Activity

Although the evidence for a relationship between LDL oxidation and the risk of ischemic heart disease and CVD is not fully established, LDL oxidation is now recognized as representing an important early event in the development of cardiovascular diseases. Oxidised LDL acts as a trigger to initiate endothelial inflammation leading to atherosclerosis and vascular thrombosis (heart attack and stroke) [1]. It was proposed that carotenoids may work by inhibiting cholesterol synthesis through the regulation of 3-hydroxy-3-methylglutaryl coenzyme a (HMGCoA) reductase [38]. Early *in vitro* studies of LDL oxidation showed that β-carotene carried in LDL is oxidized prior to the onset of oxidation of LDL polyunsaturated fatty acids, suggesting a possible role in delaying the onset of LDL oxidation [48]. On copper-mediated oxidation of the LDL, the carotenoids were destroyed before substantial amounts of lipid peroxidation products were formed, providing further evidence that these pigments may be working as antioxidants [49]. β-Carotene reacts with peroxyl radicals to give a carbon-centered carotenyl radical which, is similar to lipid free radical, in the presence of oxygen produces β-carotene peroxyl radical, so that chain propagation may occur [50]. Carotenoids have been shown to inhibit *in vivo* lipid peroxidation processes, by which the presence of carotenoids in cell membranes is essential to act as stabilizing elements of these structures [51]. Several authors have published that daily dietary β-carotene supplementation in mammals led to decreased plasma levels of total lipids, cholesterol and triglycerides. In a coculture model of the arterial wall, Dwyer *et al*. [52] found lutein to be highly effective in reducing oxidation of low density lipoproteins (LDL) and inhibiting the inflammatory response of monocytes to LDL trapped in the artery wall. They also found that dietary supplementation with lutein in two mouse models (apoE-null mice and LDL receptor-null mice) reduced plasma lipid hydroperoxides and the size of aortic lesions [52]. With *in vitro* experiments of human LDL, lutein and zeaxanthin have been shown to act as scavengers of peroxynitrite radicals [53], the product of the reaction between nitric oxide and superoxide. Further, Fuhrman and team [37] showed that the addition of lycopene to macrophage cell lines decreased cholesterol synthesis and increased LDL receptors. Incubation with lycopene *in vitro* resulted in a 73% decrease in cholesterol synthesis, which was greater than that achieved with β-carotene. Epidemiological evidence suggests that a high dietary intake of β-carotene decreases the risk for atherosclerotic vascular disease, raising the possibility that lipid-soluble antioxidants slow vascular disease by protecting LDL from oxidation. All *trans*-β-carotene inhibits atherosclerosis in hypercholesterolemic rabbits, possibly via stereospecific interactions with retinoic acid receptors in the artery wall [54].

RETRACTED

### 5.3. Antiinflammatory Activity

The NF-κB inflammatory pathway has been shown to be partially regulated by ROS and has been implicated in various forms of CVD. It is now well recognized that atherosclerosis is an inflammatory disease [55], and there is some evidence to suggest that the beneficial effects of lycopene may result from modulation of inflammatory responses. Lycopene inhibited LPS-induced production of nitric oxide (NO) and interleukin-6 (IL-6) with decreased mRNAs of inducible nitric oxide synthase and IL-6 but had no effect on TNF-α. Further study showed that lycopene also inhibited LPS-induced IκB phosphorylation, IκB degradation, and NF-κB translocation. Moreover, lycopene blocked the phosphorylation of ERK1/2 and p38 MAP kinase but not c-Jun NH_2_-terminal kinase [56]. Riso *et al*. [57] have reported that concentrations of the proinflammatory cytokine tumor necrosis factor-α (TNF-α) in the blood of healthy volunteers were decreased after dietary supplementation with a tomato-based drink. Napolitano *et al.* [58] showed that lycopene may reduce macrophage foam cell formation in response to modified LDL by decreasing lipid synthesis in the cells and down regulating the activity and expression of SR-A. These potentially beneficial effects, however, are accompanied by a marked decrease in the secretion of the anti-inflammatory cytokine IL-10, resulting in an increase in the proinflammatory profile of macrophage cytokine release. Lutein exerts potent antioxidant and anti-inflammatory effects in aortic tissue that may protect against development of atherosclerosis in guinea pigs [59]. Inflammatory mediators such as TNF-α and interleukins IL-1β, and IL-8, enhance binding of low-density lipoprotein (LDL) to endothelium and upregulate expression of leukocyte adhesion molecules on endothelium during atherogenesis. Another study examined the effects of different levels of dietary lutein and fat on LPS-induced iNOS mRNA levels in chicken macrophages. It was concluded in the study that lutein and fat or EPA act through the PPARγ and RXR pathway to change iNOS expression, and that this effect is dependent on the dose of lutein and fat or EPA [60]. 

RETRACTED

Several studies have suggested an anti-inflammatory response of lycopene. Investigations on the effect of lycopene on inflammation using oil-induced ear edema in male Kingming mice, a common screening method for determining anti-inflammatory activity are impressive [61]. Lycopene, given as tomato oleoresin, was most effective against inflammation at a dose of 0.5 g/kg body weight (*p* < 0.05). Interestingly, the inhibitory effects that occurred with a dose of 0.1 g lycopene/kg body weight were similar to those in the control group using the anti-inflammatory drug amoxicillin at the same dosage. Ohgami *et al*. [62] demonstrated multiple effects of intravenous astaxanthin administration in a uveitis model in rats, including anti-inflammatory [reductions in levels of nitric oxide (NO), tumor necrosis factor alpha (TNF-α), and prostaglandin E2 (PGE2)] and direct enzyme-inhibiting activity (against inducible nitric oxide synthase, iNOS). Another pathway in which astaxanthin combats inflammation is through inhibition of the cyclooxygenase enzymes (Cox-1 and Cox-2). In one experiment done with mice and also *in-vitro*, astaxanthin was shown to suppress TNF-α, PGE-2, IL-1β, NO as well as the Cox-2 enzyme and nuclear factor kappa-B [63]. 

## 6. Role on Endothelial Function

An imbalance of reduced production of NO and increased production of reactive oxygen species may be involved in impaired endothelium-dependent vasodilation in patients with cardiovascular risk factors and diseases. In the vascular endothelium, the free radical NO• is produced from arginine by nitric oxide synthase (NOS), converting the substrate L-arginine to L-citrulline:



The reaction requires calmodulin, NADPH and tetrahydrobiopterin (BH4) as cofactors. Under normal conditions, NO• is protective against adhesion of platelets and leucocytes, anti-inflammatory, anti-proliferative and regulates the expression and synthesis of extracellular matrix proteins.

It inhibits redox sensitive transcription factor, NFκβ expression through its binding with IKβ, linked to a number of diseases which shorten life. Oxidative damage to cholesterol component of the low-density lipoprotein (LDL) leads to oxidised LDL by a series of consecutive events. This induces endothelial dysfunction, which promotes inflammation during atherosclerosis [64]. Carotenoids and vitamins could have an antioxidant-mediated tempering influence on endothelial function and inflammation, thereby reducing the risk of atherosclerosis [65]. Martin *et al*. [66] tested carotenoid effects on vascular endothelium using human aortic endothelial cell cultures. Preincubation of lycopene resulted in a 13% decreased expression of the vascular cell adhesion molecule, a molecule present on activated endothelial tissues that aids in the recruitment of leukocytes. Enhanced production of tissue factor has been linked to development of cardiovascular disease due to endothelial activation, resulting in thrombosis of blood vessels. Akt-specific inhibitor reversed the inhibitory effect of carotenoids on tissue factor activity, indicating that carotenoids enhanced phosphorylation of Akt and suppressed tissue factor activity in endothelial cells by this mechanism [67]. 

RETRACTED

**Figure 2:** Schematic representation of carotenoids’ action on CVD.

## 7. Influence on Gap Junction Communication

Gap junction proteins called connexins mediate gap junction intercellular communication (GJC) and are a group of ≥20 highly conserved proteins with developmental and tissue-specific expression patterns. GJC allows the direct transmission among neighboring cells of ions, small hydrophilic metabolites, and messengers <1–2 kDa in size. GJC play an important role in normal development and physiology, with a loss of function implicated in various human diseases and pathologies. In the heart, electrical activation of the myocardium is necessary to produce effective pumping of blood and depends on the orderly coordinated spatial and temporal transfer of current (ions) from one cell to another [68]. In normal ventricular myocytes, this is accomplished through extensive cell-cell coupling via gap junctions. Cells have the capacity to rapidly regulate the function (posttranslational regulation), quantity (transcriptional regulation), and composition (assembly regulation) of connexins within the gap junctional structures to accommodate physiologic demands for altered cell-cell communication. Specifically, connexin 43 is the most ubiquitously expressed connexin in tissues and is essential for normal cardiac function and contraction. There has been considerable interest in the increase in gap junction communication (GJC) with carotenoids, especially lycopene, as it relates to cancer [69]. Optimal communication between endothelial cells in the artery walls is also desirable; this enhancement of GJC by lycopene may help maintain an intact and healthy endothelial surface of arteries. A well-established role of carotenoids as modulators of connexin 43 production and maintenance and/or restoration of gap junctional communication in mammals [70], suggest a multi-factorial influence of astaxanthin in cardioprotection. Several carotenoids have been shown to upregulate connexin 43 protein levels and GJC [71]. 

RETRACTED

## 8. Attenuation of Ischemia-Reperfusion Injury

Ischemia-reperfusion (I/R) injury is a complex phenomenon, generally attributed to the additional damage produced by reintroduction of oxygenated blood flow to a previously ischemic area. It is well established that cell death during (I/R) occurs via necrotic and apoptotic pathways [72] causing much damage to the heart. It has been shown that the mitogen-activated protein kinases (MAPKs), PKB/Akt and the NO-cGMP all play vital roles in ischemia/reperfusion injury in the heart. Hence, two teams worked on the role of red palm oil (RPO), carotenoid rich oil on ischemic reperfusion injury. From the results of the two teams it is evident that two pathways may play a role in the protection induced by RPO against ischemia/reperfusion injury [73,74]. The results of Esterhuyse *et al*. show that protection may occur during ischemia and that NO-cGMP may be involved. Engelbrecht *et al*. on the other hand, argue for a role of the PKB/Akt and the MAP kinases pathways in the cardioprotective effects of RPO during reperfusion. Similarly, cardioprotection and myocardial salvage by a disodium disuccinate astaxanthin derivative, *Cardax *was studied. Significant myocardial salvage is reported for the first time in that study for a novel carotenoid derivative which generates non-esterified, free astaxanthin after parenteral administration *in vivo* [75]. The mechanism(s) of action of carotenoids, and in particular astaxanthin, in cardioprotection have not been well characterized. However, Aoi and members of his lab identified that astaxanthin limits exercise-induced skeletal and cardiac muscle damage in mice [76]. It is also demonstrated that there is excellent accumulation of non-esterified, free astaxanthin in rodent myocardium after chronic oral administration of esterified, natural source of astaxanthin [77]. A dose-dependent cardioprotective effect was seen in their ROS mediated strenuous exercise injury model, with antioxidant and anti-inflammatory [*i.e.*, reduction of tissue myeloperoxidase (MPO) levels] effects observed in that seminal study. Lutein inhibited LPS- and H_2_O_2_-induced increases in phosphatidylinositol 3-kinase (PI3K) activity, PTEN inactivation, NF-κB-inducing kinase (NIK), and Akt phosphorylation, which are all upstream of IκB kinase (IKK) activation, but did not affect the interaction between Toll-like receptor 4 and MyD88 and the activation of mitogen-activated protein kinases. The study suggested that H_2_O_2_ modulates IKK-dependent NF-κB activation by promoting the redox-sensitive activation of the PI3K/PTEN/Akt and NIK/IKK pathways [78]. (I/R) causes cardiomyocyte death by activating death signals and/or inhibiting survival signals by redox signaling pathways [79]. The ability of lycopene in inhibiting IL-8 production, NF-kB/p65 nuclear translocation, and redox signalling and in increasing PPARγ expression was also found in isolated rat alveolar macrophages exposed to cigarette smoking extract [80].

RETRACTED

## 9. Conclusions

More and more evidence indicates that a proper balance between oxidants and antioxidants is involved in maintaining health and longevity and that altering this balance in favor of oxidants may result in pathological responses causing functional disorders and disease. Epidemiologic research on nutrition demonstrates that those who consume higher amounts of fruits and vegetables tend to have comparatively lower rates of heart and vascular diseases, including coronary heart disease and stroke. Short-term dietary intervention trials suggest that diets rich in fruit and vegetable intake lead to improvements in coronary risk factors and reduce cardiovascular mortality. Carotenoids are abundant, plant-derived, fat-soluble pigments that can function as antioxidants. Although more than 600 carotenoids have been identified, the majority of research in nutrition has focused on the five most common carotenoids: α-carotene, β-carotene, lycopene, lutein/zeaxanthin, and β-cryptoxanthin. Carotenoids may prevent heart and vascular disease in a number of ways as discussed earlier and summarized in Figure 2. For these reasons, carotenoids from plants may represent one plausible mechanism by which fruits and vegetables reduce the risk of CVD.

Historically, carotenoids have been known to have important beneficial properties for human health. Their biological role in the prevention and perhaps the treatment of heart and vascular diseases is now being studied and understood. Epidemiological and other population studies have shown the importance of these phytochemicals in the prevention of human diseases. *In vitro *and animal studies have tested the hypothesis generated from the epidemiological observations. Although some human clinical trials are beginning to be undertaken there is a great need for well-designed human intervention studies that take into consideration study designs including subject selection, end point measurements and the levels of carotenoids being tested. It is only through such studies that our understanding of the important role played by carotenoids will be enhanced and help us develop complementary strategies for the prevention, treatment and management of diseases.
